# Study on the Expression of lncRNA ATB and Nek9 in Breast Cancer Patients Based on Q-PCR Technology and Its Relationship with the Disease

**DOI:** 10.1155/2022/2634080

**Published:** 2022-07-14

**Authors:** Zhu Zhaoyu, Xiong Huanyu, Zhao Yajie, Dong Ziyu, Liu Hui, Shi Feng

**Affiliations:** ^1^Xinyang Vocational and Technical College, Xinyang 464000, China; ^2^Department of Image, The Affiliated Hospital of Xinyang Vocational and Technical College, Xinyang 464000, China; ^3^Department of Oncology, The Affiliated Hospital of Xinyang Vocational and Technical College, Xinyang 464000, China

## Abstract

To reveal the relationship between the expression and disease progression, the expression of long noncoding RNA ATB (lncRNA ATB) and related protein kinase 9 (Nek 9) in serum of breast cancer patients by real-time fluorescence quantitative PCR (Q-PCR) is analyzed. The patients treated in our hospital from April 2021 to February 2022 are selected and grouped into several groups. Among them, 73 patients diagnosed with breast cancer and 44 patients with benign breast disease are divided into groups A and B, respectively. In addition, 50 healthy subjects are chosen for group C. The expressions of lncRNA ATB and Nek9 in serum of patients are detected by Q-PCR, and the relationship between different pathological parameters and lncRNA ATB and Nek9 in group A is analyzed. Spearman correlation coefficient is used to evaluate the correlation between lncRNA ATB and Nek9 and disease. The experimental results show that lncRNA ATB and Nek9 in 3 groups are significantly different, and group A> group B> group C (all *P* < 0.05). The expression of lncRNA ATB and Nek9 is closely associated with lymph node metastasis and TNM stage in breast cancer patients (*P* < 0.05). Besides, the Spearman correlation coefficient shows that lncRNA ATB and Nek9 are positively correlated with breast cancer incidence (*P* < 0.05). It is evident that lncRNA ATB and Nek9 are expressed at high levels in breast cancer patients and are positively correlated with the occurrence and development of the disease.

## 1. Introduction

Breast cancer is one of the most common malignant tumors in women. The incidence rate of cancer in women is high, accounting for about 10% of all tumors. Global data show that the replacement of breast cancer has a younger trend, and its incidence rate is also increasing year by year [1]. Because the clinical manifestations of most breast cancer are not specific, most women are in advanced stage when they are diagnosed with breast cancer. This leads to poor prognosis and high mortality, which seriously threatens women's life, health, and safety [2]. At present, the commonly used serum markers in clinics mainly include CA153 and HER2 breast cancer. Although it has a certain value in the early diagnosis of breast cancer, its specificity is relatively low, which is easy to lead to misdiagnosis and missed diagnosis in clinical phenomena. Therefore, seeking a serum marker with high specificity and sensitivity is of great significance for the early diagnosis and prevention of breast cancer [3]. Gene mutation and abnormal regulation are often related to the occurrence and development of tumors. At present, breast cancer-related genes, including many oncogenes, tumor suppressor genes, and genetic susceptibility genes, have been proved to be closely related to the biological properties of breast cancer. Their expression or mutations have a predictive value for chemotherapy, endocrine therapy, and targeted therapy and affect the prognosis of patients. As the expression of long noncoding RNA (lncRNA) is involved in transcriptional activation, chromosome modification, and other functions, its horizontal expression exerts varying degrees of influence on the biological behavior of tumors. LncRNA ATB is a factor abnormally expressed in a variety of malignant tumor tissues in recent years. It is involved in the development of malignant tumors of the digestive tract and urinary system [4]. Never gene-related kinase 9 (Nek9) in mitosis is a member of the NIMA family and participates in mitosis. Nek9 participates in g^2^/m transition and regulates microtubule movement and chromosome segregation. However, there are relatively few studies on the relationship between lncRNA ATB expression in breast cancer patients and the progression of breast cancer [5]. Studying the mechanism of invasion and metastasis of breast cancer is very important for accurately evaluating the prognosis of breast cancer and finding new therapeutic targets. Therefore, it is necessary to use real-time fluorescence quantitative PCR (Q-PCR) to detect the expression of lncRNA ATB and Nek9 in breast cancer patients and further analyze the expression of these two markers in breast cancer patients.

This study is organized as follows: Section 2 discusses the related work, and the detection method and statistical treatment are introduced in Section 3.  Section 4 gives the comparative results and analysis. Some concluding remarks are made in Section 5.

## 2. Related Work

LncRNA ATB is a 2.4 kb long noncoding RNA located on human chromosome 14 [6]. At present, it has been found that it is the first RNA that can activate transforming growth factors and has abnormal expression in a variety of tumors, which can promote the occurrence and development of tumor diseases [7]. As a member of the NIMA family, Nek9 plays an important role in hammer assembly and centrosome separation control. At the same time, it has been proved that mutations in other members of the family can lead to the development of cancer. However, the role and mechanism of Nek9 in tumor cells have not been clearly described [8]. Therefore, the levels of lncRNA ATB and Nek9 in patients with breast cancer were detected by Q-PCR, and their relationship with disease development was analyzed. Exploring the specific mechanism of the above factors in breast cancer will provide effective markers for the early diagnosis of breast cancer. In addition, it can provide new molecular targets for the treatment of breast cancer.

The expression levels of lncRNA ATB and Nek9 in breast cancer patients may be positively correlated with the development of the disease and closely correlated with lymphatic metastasis and TNM stage of breast cancer. By analyzing the related mechanisms, Lu et al. [9] believed that lncRNA ATB, as a competitive endogenous RNA, can influence the expression of downstream target genes through competitive binding with miRNA and promote the proliferation of breast cancer and other malignant tumors. Moreover, the expression of miR-200c can be inhibited by binding to miR-200c binding sites to further promote the growth of breast cancer cells, and the expression levels of miR-200c target genes ZEB1 and ZEB2 can be increased, while the highly expressed ZEB1 and ZEB2 can promote the epithelial-mesenchymal transition of cancer cells. Furthermore, promote the progress of the disease [10]. In addition, the higher the TNM stage is, the higher the expression of lncRNA ATB will be. It also suggested the involvement and deterioration of lncRNA ATB, and the expression of lncRNA ATB in breast cancer patients with lymphatic metastasis is higher than that in nonlymph nodes. It indicated that lncRNA ATB is involved in the invasion and metastasis of cancer cells. It is shown that lncRNA ATB promotes the invasion and metastasis of cancer cells in breast cancer patients, participates in the deterioration of the disease, and jointly promotes the further development of the disease [11]. The downregulation of lncRNA ATB breast cancer cells can significantly reduce the mobility of cells compared with the negative control group, resulting in the loss of adhesion and connection function of epithelial cells and the acquisition of mesenchymal cell characteristics [12]. At the same time, the increased expression levels of E-cadherin and vimentin can further promote the invasion and migration of cancer cells and aggravate the disease.

The Nek family is involved in cell mitosis in the body and includes Nek9 and other 11 members. Currently, the mechanism and function of most members have not been clearly described. Nek2 can regulate the ERK/MAPK pathway, thus promoting the proliferation of gastric cancer cells and the development of gastric cancer. In addition, some scholars pointed out that Nek2 and Nek9 jointly promote the development of tumor diseases, but the mechanism of action of Nek9 in breast cancer is not clear yet [13]. In this study, Nek9 is highly expressed in breast cancer patients and is closely related to breast cancer development, lymphatic metastasis, and TNM staging, suggesting that Nek9, as an essential substance for cell mitosis and maintenance of normal proliferation, can be activated and phosphorylated in cell mitosis to combine with Nek6 and 7 [14]. Xu et al. [15] also pointed out that in normal cells, Nek9 has the effect to maintain normal cell division, the appreciation to a certain extent, and can inhibit tumor cells. However, for the Nek9 silent group, tumor cells lack the Nek9 effect on regulating cell mitosis key points, can cause tumor cell of appreciation, and further promote the development of illness [16–19]. However, the specific mechanism of its action needs to be further elaborated by more basic research.

## 3. Detection Method and Statistical Treatment

### 3.1. Detection Method

A retrospective analysis is performed on 73 patients diagnosed with breast cancer in our hospital from April 2021 to February 2022 as group A, 44 patients with benign breast disease as group B, and 50 healthy people as group C. The comparison of baseline data among each group is given in Table 1, indicating comparability (*P* > 0.05). The clinical data obtained in this study will only be used for research purposes, not for other purposes.

The principles stipulated in the inclusion criteria are as follows: meet the clinical diagnostic criteria for breast cancer [6], there was no distant organ metastasis at the time of inclusion, complete clinical data and general information [20], and signed informed consent. In addition, the exclusion criteria stipulated the following principles: patients with other tumor lesions [21], lack of clinical data [22], patients with mental illness cannot obtain a high degree of research coordination [23], and congenital immunodeficiency [24].

The specific detection procedures are as follows: 5 ml peripheral blood is taken from patients in both groups on an empty stomach in the morning and centrifuged at 3500 r/min (centrifuge radius: 13.5 cm) for 10 min. After centrifugation, upper serum is separated and placed in a refrigerator at −70°C for detection. The serum to be measured is taken and total RNA is extracted by the TRIzol method. 0.2 mL chloroform is added to every 1 mL of TRIzol reagent lysis sample, and the samples are vigorously oscillated for 15 s, incubated for 3 min at 15–30°C, and centrifuged at 12 000 RPM at 4°C for 15 min. After centrifugation, the mixed liquid will be divided into a lower layer of red phenol-chloroform phase, an intermediate layer, and a colorless water phase. Transfer the upper layer of the aqueous phase to a clean RNA-free centrifuge tube. Isopropyl alcohol is added to the mix to precipitate the RNA. After mixing, the RNA is incubated at 15–30°C for 10 min and centrifuged at 12000 rpm at 4°C for 10 min. The supernatant is removed, and at least 1 ml of 75% ethanol is added to every 1 ml of TRIzol lysed sample and then centrifuged at 7000 rpm at 4°C for 5 min. Most of the ethanol solution is carefully sucked away, and the RNA is precipitated and dried in air at room temperature for 5–10 minutes. To dissolve RNA, 40 ul of water without RNA enzyme is first added with a gun several times to make it completely dissolved. The RNA solution obtained is stored at −80°C for later use. Its integrity and purity are tested at 4°C, and the ratio of A260/A280 of RNA solution is RNA purity, ranging from 1.8 to 2.1. Reverse transcription is performed at 42°C for 60 min and 70°C for 10 min and preserved at 4°C. The amplified products are analyzed by 3 G/DL agarose gel electrophoresis and stained with anthocyanin ethidium bromide. The Ct values are obtained by gel imager, and the changes are expressed as *δ* Ct [18]. Using GAPDH as an internal reference, the primer sequence is 5′-GGGAGCCAAAAGGGTCAT-3′ upstream and 5′-GAGtCCTTCCACGATACCA-3′ downstream, and the length of the amplified product is 720 bp. LncRNA ATB upstream primer 5′-TACAACCACTGCACTACCTG-3′, downstream primer 5′-TGGAATGCTTGAAGgCTGCT-3′, Nek9 upstream primer 5′-CCTGGATCCTGTTGACACCC-3′, downstream 5′-ACAGGGGAAACGCAGGATTT-3′, and the relative expression levels of lncRNA ATB and Nek9 are calculated by the 2^−ΔΔCt^ method [19]. Table 1 provides the comparison of baseline data. Reagents and instruments required for the test are given in Table 2.

### 3.2. Statistical Treatment

All data during the study are collected and sorted out and then put into SPSS 22.0 for statistical processing. If the measurement data followed normal distribution and homogeneity of variance, they are expressed as mean ± standard deviation (*‾x* ± *s*), and intergroup differences are performed by the independent sample *t*-test, the intragroup comparison is performed by the paired *t*-test and intergroup F test. Count data are represented by (%), and the differences between groups are tested by *x*^*2*^. Spearman correlation coefficient is used to analyze the correlation between lncRNA ATB and Nek9 and breast cancer incidence. ROC curve analysis of combined detection for early diagnosis of breast cancer will be conducted. All the above data are at *P* < 0.05, and the differences among the data are statistically significant.

## 4. Result, Analysis, and Discussion

### 4.1. Comparison of lncRNA ATB and Nek9 Expression Differences

There are significant differences in lncRNA ATB and Nek9 among the three groups, and group A> group B> group C (all *P* < 0.05), as given in Table 3 and Figure 1.

### 4.2. Analysis of the Relationship between Different Pathological Parameters and lncRNA ATB Expression in Breast Cancer Patients

LncRNA ATB expression is associated with lymph node metastasis and TNM stage in breast cancer patients (*P* < 0.05), but not with age or tumor size (*P* > 0.05), as given in Table 4. The results demonstrate that the expression levels of lncRNA ATB and Nek9 in breast cancer patients are significantly higher than those in benign breast lesions and normal controls, which are positively correlated with the development of the disease and closely correlated with lymphatic metastasis and TNM stage of breast cancer (all *P* < 0.05).

### 4.3. Analysis of the Relationship between Nek9 Expression of Different Pathological Parameters in Breast Cancer Patients

Nek9 expression is associated with lymph node metastasis and TNM stage in breast cancer patients (*P* < 0.05), but not with age or tumor size (*P* > 0.05), as given in Table 5.

### 4.4. Spearman Correlation Coefficient Analysis of the Relationship between lncRNA ATB and Nek9 and the Incidence of Breast Cancer

Spearman's correlation coefficient showed that lncRNA ATB and Nek9 are positively correlated with the incidence of breast cancer (both *P* < 0.05), as given in Table 6.

### 4.5. ROC Curve Evaluation of Combined Detection of lncRNA ATB and Nek9 for the Diagnosis of Breast Cancer

Since both lncRNA ATB and Nek9 are expressed specifically in breast cancer patients, this study analyzed the diagnostic efficacy of the combined detection of the two indicators by drawing ROC. The diagnostic efficiency of each indicator is given in Table 7. ROC curve shows that the detection rate of combined detection for breast cancer is significantly higher than that of single detection, suggesting that combined detection of lncRNA ATB and Nek9 has a high diagnostic value for breast cancer, as shown in Figure 2. ROC curve shows that lncRNA ATB combined with Nek9 had high diagnostic efficacy for breast cancer, and its area under the curve is significantly higher than that of any single test, with a sensitivity of 87.70% and specificity of 82.10%. It can be observed that the area under the curve in the combined detection is significantly higher than that of the single detection, indicating that the above two biological indicators play a driving role in breast cancer. Therefore, it has a high application value for early diagnosis of such diseases.

## 5. Conclusions

In this study, the expression of long noncoding RNA ATB (lncRNA ATB) and related protein kinase 9 (Nek 9) in serum of breast cancer patients by real-time fluorescence quantitative PCR (Q-PCR) is analyzed to explore the relationship between the expression and disease progression. The experimental results reveal that lncRNA ATB and Nek9 are highly expressed in breast cancer patients, are significantly associated with lymphatic metastasis and TNM staging of breast cancer, and promote the development of breast cancer. Combined detection can improve the efficiency of early diagnosis. However, there are relatively few clinical studies on the pathogenesis of lncRNA ATB and Nek9 in breast cancer. In the future, we will conduct more basic research and clinical experiment to further validate the findings.

## Figures and Tables

**Figure 1:** Comparison of lncRNA ATB and Nek9 expression differences.

**Figure 2:** ROC curve evaluation of combined detection of lncRNA ATB and Nek9 for the diagnosis of breast cancer.

**Table 1:** Comparison of baseline data.

Item	Number	Age	BMI (kg/m^2^)
Group A	73	43.32 ± 6.43	23.32 ± 2.55
Group B	44	43.19 ± 6.38	23.28 ± 2.28
Group C	50	42.97 ± 6.52	23.41 ± 2.31
*F*		5.563	5.391
*P*		0.748	0.693

**Table 2:** Reagents and instruments.

Reagent/instrument	Place of origin	Manufacturer
TRIzol	American	Invitrogen
Centrifuge	American	Themor
Chloroform	China	Chengdu Kelon Chemical Reagent Factory
Ethyl alcohol	China	Chengdu Kelon Chemical Reagent Factory
PCR amplifier	Switzerland	Roche
Internal primers	China	Shanghai Shenggong Bioengineering Co., Ltd.

**Table 3:** Comparison of lncRNA ATB and Nek9 expression levels.

Item	Number	lncRNA ATB	Nek9
Group A	73	1.85 ± 0.24	0.41 ± 0.08
Group B	44	1.17 ± 0.27	0.24 ± 0.05
Group C	50	0.83 ± 0.21	0.12 ± 0.04
*F*		0.665	0.139
*P*		0.051	0.053

**Table 4:** Relationship between pathological parameters of breast cancer and lncRNA ATB.

Clinicopathological parameters	*n*	lncRNA ATB	*t*	*P*
Age (years)			−0.335	0.739
＜45	36	1.79 ± 0.25		
≥45	37	1.81 ± 0.26		

Tumor diameter (cm)			0.177	0.860
≤2	42	1.82 ± 0.23		
＞2	31	1.81 ± 0.25		

Lymph node metastasis			5.475	<0.001
Y	41	1.96 ± 0.28		
N	32	1.62 ± 0.24		

TNM staging			−2.843	0.006
I-II	35	1.71 ± 0.25		
III-IV	38	1.88 ± 0.26		

**Table 5:** Relationship between pathological parameters of breast cancer and Nek9.

Clinicopathological parameters	*n*	Nek9	*t*	*P*
Age (years)			0.449	0.655
＜45	36	0.40 ± 0.09		
≥45	37	0.39 ± 0.10		

Tumor diameter (cm)			−1.001	0.320
≤2	42	0.39 ± 0.08		
＞2	31	0.41 ± 0.09		

Lymph node metastasis			5.847	<0.001
Y	41	0.42 ± 0.08		
N	32	0.32 ± 0.06		

Tumor staging			−6.245	<0.001
I-II	35	0.30 ± 0.07		
III-IV	38	0.41 ± 0.08		

**Table 6:** Correlation analysis.

Item	Breast cancer	
	*r*	*P*
lncRNA ATB	0.782	＜0.001
Nek9	0.766	＜0.001

**Table 7:** Diagnostic performance table.

Detection method	95% CI	Sensitivity (%)	Specificity (%)	AUC	Cutoff value
Joint detection	0.882–0.981	87.70	82.10	0.931	—
lncRNA ATB	0.672–0.829	78.30	78.20	0.751	
Nek9	0.512–0.684	61.20	62.20	0.598	

## Data Availability

The data used to support the findings of this study are available from the corresponding author upon request.
